# The Effects of Age and Latent Cytomegalovirus Infection on NK-Cell Phenotype and Exercise Responsiveness in Man

**DOI:** 10.1155/2015/979645

**Published:** 2015-10-25

**Authors:** Austin B. Bigley, Guillaume Spielmann, Nadia Agha, Richard J. Simpson

**Affiliations:** Laboratory of Integrated Physiology, Department of Health and Human Performance, University of Houston, 3855 Holman Street, Houston, TX 77204, USA

## Abstract

The redeployment of NK-cells in response to an acute bout of exercise is thought to be an integral component of the “fight-or-flight” response, preparing the body for potential injury or infection. We showed previously that CMV seropositivity impairs the redeployment of NK-cells with exercise in the young. In the current study, we examined the effect of aging on the redeployment of NK-cells with exercise in the context of CMV. We show here that CMV blunts the exercise-induced redeployment of NK-cells in both younger (23–39 yrs) and older (50–64 yrs) subjects with older CMV^neg^ subjects showing the largest postexercise mobilization and 1 h postexercise egress of NK-cells. The blunted exercise response in CMV^pos^ individuals was associated with a decreased relative redeployment of the CD158a+ and CD57+ NK-cell subsets in younger and older individuals. In addition, we show that aging is associated with a CMV-independent increase in the proportion of NK-cells expressing the terminal differentiation marker CD57, while CMV is associated with an age-dependent decrease in the proportion of NK-cells expressing the inhibitory receptors KLRG1 (in the younger group) and CD158a (in the older group). Collectively, these data suggest that CMV may decrease NK-cell mediated immunosurveillance after exercise in both younger and older individuals.

## 1. Introduction

The rapid redeployment of NK-cells between the tissues and the peripheral circulation is an archetypal feature of the acute stress response. The response can be evoked using acute bouts of dynamic exercise [1, 2], laboratory-based psychological stress tasks [3], or beta-agonist (i.e., epinephrine) infusion [4] and is often considered to be an accurate representation of an organism's ability to mount an effective immune response during fight-or-flight scenarios when tissue injury and infection are likely to occur. Acute exercise is associated with increased plasma levels of stress hormones including the catecholamines epinephrine and norepinephrine [5], which interact with *β*-adrenergic receptors (*β*-AR) on the surface of lymphocytes. NK-cells express more *β*-AR than other lymphocytes [6] and, as a result, they are the most responsive lymphocyte subset to exercise [7, 8] and catecholamines [4, 9].

Cytomegalovirus (CMV) is a prevalent beta herpesvirus infecting 50–80% of the US population [10, 11]. We have shown that prior exposure to CMV profoundly impacts the redistribution of lymphocytes to an acute exercise bout. While those with CMV have an augmented redeployment of CD8+ T-cells [12, 13] and *γδ* T-cells [14], NK-cell mobilization is dramatically impaired [15]. This blunted NK-cell response appears to be attributable to a CMV-induced accumulation of specific NK-cell subsets that have a lower expression of *β*2-AR and an impaired ability to produce cyclic AMP in response to* in vitro* stimulation with the *β*-agonist isoproterenol [16]. Moreover, those with CMV fail to exhibit exercise-induced enhancements in NK-cell function, indicating that CMV may compromise NK-cell mediated immunosurveillance after an acute bout of strenuous exercise [16].

In addition to infection history, aging is known to have a profound impact on the cellular response to acute stress and exercise [17]; however, studies investigating the effects of aging on NK-cell exercise responsiveness are lacking [18]. While aging has been reported to have no effect on NK-cell mobilization with exercise [19, 20], it is known to increase the proportion of CD56dim/KIR+/CD57+ NK-cells [19, 21, 22], a subset we have previously shown to be preferentially mobilized by exercise [23]. In addition, several of the phenotypic hallmarks of aging overlap with those associated with latent CMV infection in the young including upregulation of CD57 [19, 24, 25] and downregulation of KLRG1 [15, 26]. Despite CMV prevalence increasing with age [11], previous studies have compared NK-cell responses between young and old exercisers without accounting for this confounding variable [19, 20]. We showed recently that CMV was associated with enhanced redeployment of CD8+ T-cells regardless of age [13], while, conversely, aging impairs the redeployment of *γδ* T-cells independently of CMV [14]. However, no study to our knowledge has compared NK-cell responses to a single bout of exercise between different age groups while controlling for CMV serostatus. Given that CMV prevalence increases with age and many of the effects of CMV mirror those attributable to aging, it is important to resolve the effects of age and CMV infection on the frequency and exercise responsiveness of distinct NK-cell subsets.

The aim of this study was to determine if latent CMV infection blunts the redeployment of NK-cells to a single exercise bout in older individuals as it does in the young [15] and to delineate the effects of age and CMV on the redeployment of discrete NK-cell subsets. We show here that CMV has a potent blunting effect on exercise-induced NK-cell mobilization in both younger (23–39 yrs) and older (50–64 yrs) subjects with the greatest mobilization being seen in the CMV^neg^ older group. This blunting effect of CMV was most pronounced with the CD158a+ and CD57+ NK-cell subsets regardless of age.

## 2. Materials and Methods

### 2.1. Participants

40 healthy adult males (age: 23–64 years) participated in this study. The exclusion criteria of this study required that participants avoid smoking, medication/supplements, or infection within 6 weeks of the experiment. Oral and written information regarding the risks and requirements of the study were provided, after which each participant signed an informed consent affidavit. Protocol approval was granted by CPHS at the University of Houston. Participant attributes and exercise data are provided in Table 1.

### 2.2. Exercise Protocols and Blood Sampling

Maximal oxygen uptake ($\dot{V}O_{2}$ max) was estimated using the Astrand [30] submaximal cycling exercise protocol as previously described [15]. The Adams and Beam equations [29] were used to estimate the $\dot{V}O_{2}$ max and maximum power of each participant.

Participants reported to the lab following an overnight fast within 2 weeks (minimum: 2 days) of the submaximal $\dot{V}O_{2}$ max test to complete a 30 min cycling protocol. A resting intravenous blood sample was collected in 6 mL Vacutainers containing either EDTA or serum gel (BD, Franklin Lakes, NJ, USA) prior to exercise. Participants then cycled for 30 min at 80% of max power and peripheral blood samples were collected again immediately after and 1 h after exercise. Serum was frozen at −80°C until analysis (in duplicate) for CMV IgG antibodies using commercially available ELISA kits (BioCheck, Foster City, CA, USA) and a 96-well microplate reader (Molecular Devices, Sunnyvale, CA, USA).

### 2.3. Flow Cytometry

PBMCs were separated from whole blood using Histopaque per the manufacturer's instructions (Sigma-Aldrich, St. Louis, MO, USA). Aliquots of 1 × 10^6^ isolated cells were incubated for 30 minutes with 50 *μ*L of prediluted APC-conjugated anti-CD3, Alexa488-conjugated anti-KLRG1 [31] or FITC-conjugated anti-CD56, PerCP-Cy5.5-conjugated anti-CD8 or PerCP-eFluor710-conjugated anti-CD56, and PE-conjugated anti-CD57 or anti-CD158a monoclonal antibodies. All of the antibodies were purchased from eBioscience (San Diego, CA, USA) except for the anti-KLRG1 antibody that was generously provided by Dr. Hanspeter Pircher. Lymphocyte phenotype and cell count were assessed by 4-color flow cytometry using an Accuri C6 flow cytometer (Accuri, Ann Arbor, MI, USA) as previously described [15].

### 2.4. Statistical Analysis

SPSS version 22 (Chicago, IL, USA) was used for all statistical analyses. The effects of CMV and age on NK-cell phenotype, participant attributes, and exercise data were determined using a separate restricted maximum likelihood linear mixed model (LMM) including main effects for CMV serostatus and age, as well as an interaction term for CMV serostatus *∗* age. To determine the effects of CMV and age on the acute exercise response of NK-cell subsets, a LMM was built that included main effects for CMV serostatus, age, and exercise (before, after, and 1 h after), as well as interaction terms for CMV serostatus *∗* exercise and age *∗* exercise. The precise location of significant main effects was determined using Bonferroni post-hoc analysis. Independent sample *t*-tests were used to compare delta values (i.e., cells mobilized and egressed by exercise) relative to CMV serostatus and age. Statistical significance was assessed at *p* < 0.05.

## 3. Results

### 3.1. Age and CMV Have Distinct Effects on NK-Cell Phenotype

To determine the effects of age and CMV on NK-cell subsets, we evaluated NK-cell phenotype in the context of age and latent CMV infection (Figure 1). Aging increases the proportion of CD57+ NK-cells [*F*(1, 180) = 6.551, *p* < 0.01] and decreases the proportion of CD56-bright NK-cells [*F*(1, 180) = 5.363, *p* < 0.05]. The effects of age on CD57+ and CD56-bright NK-cells were CMV independent [*F*(1, 180) = 0.37, *p* = 0.554 and *F*(1, 180) = 0.022, *p* = 0.882, resp.]. While there was no overall effect of age on NK-cell CD158a expression [*F*(1, 180) = 2.581, *p* = 0.111], there was an interaction effect between CMV and age [*F*(1, 180) = 3.91, *p* < 0.05]. The proportion of CD158a+ NK-cells was lower in the CMV^pos^ older (50–64 yrs) group (*p* < 0.05). While there was no main effect of age on NK-cell KLRG1 [*F*(1, 180) = 0.154, *p* = 0.695] or CD8 expression [*F*(1, 180) = 1.904, *p* = 0.169], the proportion of KLRG1+ NK-cells was greater in the CMV^neg^ younger (23–39 yrs) group (*p* < 0.05) and the proportion of CD8+ NK-cells was greater in the CMV^neg^ older group (*p* < 0.05).

### 3.2. Latent CMV Infection Impairs the Exercise-Induced Mobilization of NK-Cells in Both Younger and Older Adults

The effects of age and CMV serostatus on the exercise response of total NK-cells and NK-cell subsets are shown in Table 2. The number of total NK-cells and all NK-cell subsets was increased immediately after exercise compared to baseline and 1 h after exercise (*p* < 0.001). There was a main effect of CMV serostatus on total NK-cell number [*F*(1, 168) = 5.652, *p* < 0.05] that was independent of age [*F*(1, 168) = 1.323, *p* = 0.252]. The main effect of CMV serostatus was the result of fewer NK-cells immediately after exercise (*p* < 0.05). There was no main effect of age on total NK-cell number [*F*(1, 168) = 2.617, *p* = 0.108]; however, the postexercise NK-cell count was greater in older relative to younger CMV^neg^ subjects (*p* < 0.05).

The exercise responsiveness of NK-cells based on CMV serostatus and age is described in Figure 2(a). CMV seropositivity was associated with a lower exercise-induced redeployment of NK-cells [*F*(2, 168) = 4.664, *p* < 0.05] that was independent of age [*F*(2, 168) = 1.037, *p* = 0.357]. Specifically, the mobilization and egress of NK-cells were greater in CMV^neg^ individuals regardless of age (*p* < 0.05) as seen in Figure 2(b). Age did not affect the redeployment of NK-cells with exercise [*F*(2, 168) = 0.587, *p* = 0.557].

Aging was associated with an increased percentage of NK-cells within the lymphocyte pool [*F*(1, 168) = 5.123, *p* = 0.025] that was dependent on CMV serostatus [*F*(1, 168) = 12.777, *p* < 0.001]. Specifically, the proportion of NK-cells was elevated in older subjects that were CMV^neg^ (*p* < 0.05) but not in those that were infected with CMV (*p* > 0.05). As with cell number, CMV seropositivity was associated with a lower proportional increase in NK-cells after exercise [*F*(2, 168) = 3.221, *p* < 0.05] that was independent of age [*F*(2, 168) = 1.258, *p* = 0.287]. Representative flow cytometry dot-plots illustrating the age-independent blunting of NK-cell exercise responsiveness in those infected with CMV are shown in Figure 2(c).

### 3.3. Latent CMV Infection Decreases the Exercise Responsiveness of CD57+ and CD158a+ NK-Cells Independently of Age

To assess the effects of age and CMV on the redeployment of NK-cell subsets with exercise, we evaluated exercise-induced changes in the proportion of NK-cell subsets in relation to age and latent CMV infection (Figure 3(a)). The proportion of CD57+ and CD158a+ NK-cells is increased immediately after exercise (*p* < 0.05). The exercise effects on NK-cell CD57 and CD158a expression were independent of CMV [*F*(2, 180) = 0.016, *p* = 0.984 and *F*(2, 180) = 0.075, *p* = 0.927, resp.] and age [*F*(2, 180) = 0.213, *p* = 0.808 and *F*(2, 180) = 0.312, *p* = 0.732, resp.]. The mobilization and egress of CD57+ and CD158a+ NK-cells were greater in CMV-seronegative subjects relative to those infected with CMV (*p* < 0.05). In addition, the proportion of CD56-bright NK-cells was increased 1 h after exercise (*p* < 0.05) independently of CMV [*F*(2, 180) = 0.059, *p* = 0.942] and age [*F*(2, 180) = 0.016, *p* = 0.984]. Exercise had no effect on NK-cell KLRG1 or CD8 expression [*F*(2, 180) = 0.404, *p* = 0.668 and *F*(2, 180) = 0.018, *p* = 0.982, resp.]. In addition, CMV serostatus did not affect the mobilization or egress of CD56-bright, KLRG1+, or CD8+ NK-cells (*p* > 0.05). Representative flow cytometry dot-plots for the coexpression of KLRG1 and CD57 in relation to exercise are shown in Figure 3(b).

## 4. Conclusions

This is the first study to examine the effects of aging and latent CMV infection on NK-cell redeployment in response to a single bout of intensity-controlled exercise. We report that latent CMV infection is associated with a blunted exercise-induced redeployment of NK-cells in both younger (23–39 yrs) and older (50–64 yrs) subjects with older CMV^neg^ subjects showing the greatest postexercise mobilization and 1 h postexercise egress of NK-cells. This blunted exercise response in CMV^pos^ individuals was associated with a decreased relative redeployment of the CD158a+ and CD57+ NK-cell subsets in both younger and older individuals. In addition, we show for the first time that the previously reported age-associated increase in the proportion of CD57+ NK-cells is independent of CMV, while the proportion of CD8+ NK-cells and the percentage of NK-cells in the lymphocyte pool are increased in older CMV^neg^ individuals only. Further, CMV is associated with an age-dependent decrease in the proportion of NK-cells expressing the inhibitory receptors KLRG1 (lower in younger CMV^pos^) and CD158a (lower in older CMV^pos^).

The redeployment of cytotoxic lymphocytes (including NK-cells) in response to an acute bout of exercise is thought to be an integral part of the “fight-or-flight” response, preparing the body for potential injury or infection [3]. We show here that CMV seropositivity is associated with a blunted redeployment of NK-cells in older subjects and that increased age is associated with a greater redeployment of NK-cells in CMV^neg^ individuals. This builds on our previous finding that latent CMV infection is associated with a blunted exercise-induced redeployment of NK-cells in the young [15]. Alternatively, it has been reported that the mobilization of CD8+ cytotoxic T-cells is greater in CMV^pos^ individuals [12] and we have shown that this CMV effect is particularly pronounced in the old [13]. Considering that there is no difference in lymphocyte mobilization between CMV^pos^ and CMV^neg^ individuals [12, 13], it appears that the effects of CMV on redeployment of cytotoxic CD8+ T-cells and NK-cells largely offset each other. Thus, it could be that postexercise immunosurveillance is tilted towards T-cell-mediated immunity in CMV^pos^ individuals and NK-cell mediated immunity in CMV^neg^ individuals with this contrast being most evident in older individuals. Given the decline in T-cell function with age [32] and the accumulation of senescent T-cells in those with CMV [33], this suggests a general decline in postexercise immunosurveillance in older CMV^pos^ individuals.

The redeployment of individual NK-cell subsets with exercise is nonuniform. We have previously reported that NK-cells expressing inhibitory KIR (such as CD158a) and the terminal differentiation marker CD57 are preferentially mobilized by exercise [23]. In the current study, we report that the mobilization of CD158a+ and CD57+ NK-cells with exercise is reduced in CMV^pos^ individuals regardless of age. We have shown earlier that CMV impairs NK-cell mobilization in response to high intensity exercise through downregulation of *β*2-AR expression on CD57+ NK-cells and impaired *β*-AR signaling in younger CMV^pos^ individuals [16]. This mechanism likely applies to older subjects as well given the similar impairment in CD57+ NK-cell exercise responsiveness between younger and older CMV^pos^ subjects. The decreased exercise-induced redeployment of CD57+ NK-cells in CMV^pos^ individuals is likely to have functional implications as CD57+ NK-cells have high cytotoxic functions, but greatly reduced proliferative capacity [34, 35]. Due to their high expression of differentiation markers [36] and their poor cytokine-driven proliferation, CD57+ NK-cells are considered to be terminally differentiated [34].

We show here that CMV and age combine to influence NK-cell phenotype in many interesting ways that have often been overlooked in the literature due to failure to recruit older CMV^neg^ individuals. For example, it has been reported in multiple studies that the proportion of CD57+ NK-cells is increased in the elderly [19, 37, 38]; however, it has been reported by Campos et al. that this aging effect is actually a CMV effect with CMV^pos^ subjects having a higher proportion of CD57+ NK-cells regardless of age [24]. The conclusions of Campos et al. are limited, however, by the lack of CMV^neg^ elderly in their cohort [24]. Our study includes older CMV^neg^ individuals and contradicts the findings of Campos et al. [24] as we show a CMV-independent increase in the proportion of CD57+ NK-cells with aging. These findings are consistent with the CMV-independent increase in the CD56dim : CD56 bright ratio with age shown here and elsewhere [21], which suggests that the accumulation of highly differentiated NK-cells is attributable to aging independently of latent CMV infection. The increased proportion of CD56dim CD57+ NK-cells in the older group likely contributes to the increased exercise-induced redeployment of NK-cells in older relative to younger CMV^neg^ individuals. One of the limitations of this study is that we did not measure CD16 expression on NK-cells. CD16 is a marker of NK-cell differentiation and it is functionally important as it plays a critical role in NK-cell mediated antibody-dependent cytotoxicity [39]. We were unable to include CD16 as a marker of differentiation because we were limited by the constraints of 4-color flow cytometry.

We report a CMV-dependent decrease in the proportion of CD158a+ NK-cells with age. There was no overall difference in the proportion of CD158a+ NK-cells between younger and older subjects; however, the proportion of CD158a+ NK-cells was decreased in CMV^pos^ older subjects. Multiple studies have reported no effect of aging on inhibitory KIR expression [38, 40, 41]; however, one study reported an increase in inhibitory KIR expression with age [22]. None of these earlier studies investigated the relationship between these aging effects and CMV infection. We also show that the proportion of KLRG1+ NK-cells is decreased in younger CMV^pos^ individuals, but there is no CMV effect in the older group and no overall aging effect either. Our current data contradict a previous report by Hayhoe et al. that aging is associated with a marked decrease in the proportion of KLRG1+ NK-cells [26]. The discrepancy between our findings and those of Hayhoe et al. [26] are likely due to different definitions of young and old between the two studies. Hayhoe et al. compared individuals older and younger than 60 years [26], while we compared individuals aged 23–39 years to individuals aged 50–64 years. In our study, we investigated aging in preelderly (less than 65 years old), otherwise healthy individuals (presymptomatic for any age-related diseases). Future studies should determine if our results regarding the effects of aging and CMV on NK-cell phenotype and exercise responsiveness apply to females and individuals over the age of 65 as well.

In addition, we show for the first time that the previously reported increase in NK-cell proportion with age [22, 24] is CMV-dependent. Specifically, the proportion of NK-cells in the peripheral lymphocyte pool is elevated in CMV^neg^ older subjects, but not older subjects with CMV. The proportion of CD8+ NK-cells is also elevated in CMV^neg^ older subjects only, which suggests a possible increase in NK-cell cytotoxicity as CD8 expression has been mechanistically linked to increased NK-cell activity [42]. On the other hand, we have reported increased baseline NK-cell activity and impaired functional responses to exercise in younger CMV^pos^ individuals [16]. Thus, future studies are needed to determine the combined effects of CMV and aging on NK-cell function before and after exercise.

In summary, latent CMV infection was associated with a marked reduction in the mobilization of NK-cells in response to exercise in both younger and older adult males with the greatest mobilization being seen in CMV^neg^ older subjects. We also show that age was associated with a CMV-independent increase in the proportion of terminally differentiated CD57+ NK-cells and that CMV was associated with an age-dependent decrease in the proportion of NK-cells expressing the inhibitory receptors KLRG1 (lower in younger group) and CD158a (lower in older group). We conclude that latent CMV infection may compromise NK-cell mediated immunosurveillance following an acute stress response in both younger and older males.

## Figures and Tables

**Figure 1:** The effects of latent CMV infection and age on the proportion of total NK-cells (% of lymphocytes) and NK-cell subsets (% of NK-cells). Values are mean ± SE. Significance is connoted by ^#^ *p* < 0.05.

**Figure 2:** Latent CMV infection impairs the exercise-induced mobilization of NK-cells in both younger and older adults. (a) shows the effect of exercise at 80% of estimated maximum power on NK-cell count based on latent CMV infection and age. (b) shows the effect of latent CMV infection and age on the mobilization and egress of NK-cells in response to an acute bout of exercise at 80% of estimated maximum power. Values are mean ± SE. Differences based on CMV serostatus and age are indicated by ^#^ *p* < 0.05 and ^∧^ *p* < 0.05, respectively. (c) displays representative flow cytometry dot-plots for the redeployment of NK-cells with exercise relative to CMV serostatus and age.

**Figure 3:** Latent CMV infection decreases the exercise responsiveness of CD57+ and CD158a+ NK-cells independently of age. (a) shows the effects of CMV and age on the redeployment of CD57+ and CD158a+ NK-cells in response to an acute bout of exercise at 80% of estimated maximum power. Values are mean ± SE. Differences based on CMV serostatus are connoted by ^#^ *p* < 0.05. (b) displays representative flow cytometry dot-plots for the coexpression of KLRG1 and CD57 before and after exercise based on latent CMV infection and age.

**Table 1:** Physical characteristics of the participants (*N*_CMV+_ = 20; *N*_CMV−_ = 20). Data are mean ± SD. CMV seronegative and CMV seropositive participants indicated by − and +, respectively. Statistical differences between younger (23–39 yrs) and older (50–64 yrs) subjects are indicated by ^#^ *p* < 0.05. CMV serostatus did not affect any of the physical characteristics (*p* > 0.05).

Characteristics	Younger (−) [*N* = 12]	Younger (+) [*N* = 12]	Older (−) [*N* = 8]	Older (+) [*N* = 8]	One-way ANOVA *F* statistic (*p* value)	
					CMV	Age
Age (years)	30.8 ± 6.4	30.0 ± 6.0	55.6 ± 3.6^#^	57.1 ± 4.1^#^	<0.1 (0.88)	163.1 (<0.001)
Height (cm)	179.4 ± 7.1	177.9 ± 5.4	178.2 ± 8.6	177.2 ± 6.3	1.3 (0.26)	0.1 (0.72)
Mass (kg)	81.2 ± 12.8	82.8 ± 12.1	79.6 ± 8.1	79.8 ± 10.2	<0.1 (0.98)	<0.1 (0.84)
BMI (kg·m^−2^)	25.1 ± 3.2	25.7 ± 4.7	24.8 ± 2.1	25.8 ± 2.7	0.5 (0.45)	<0.1 (0.90)
Maximum power (W)	241.3 ± 76.5	226.2 ± 57.0	235.7 ± 65.6	225.8 ± 38.8	0.4 (0.53)	<0.1 (0.88)
*V*O_2max_ (mL·kg^−1^·min^−1^)	39.6 ± 13.0	36.7 ± 6.3	40.7 ± 17.4	40.3 ± 7.5	0.4 (0.49)	<0.1 (0.90)
Maximum heart rate^**∗**^ (bpm)	187.7 ± 6.1	187.8 ± 5.8	164.4 ± 3.6	164.9 ± 3.7	<0.1 (0.87)	163.4 (<0.001)
Physical activity rating^a^ (0–7)	5.0 ± 2.2	5.4 ± 2.1	6.3 ± 1.0	5.6 ± 1.9	<0.1 (0.90)	3.2 (0.09)
Age-adjusted fitness score^b^ (1–5)	3.6 ± 1.8	3.1 ± 1.1	4.1 ± 1.2	3.7 ± 1.0	<0.1 (0.83)	2.2 (0.14)

*Exercise measures *						
Mean power (W)	183.6 ± 63.5	175.8 ± 61.1	181.3 ± 38.5	172.4 ± 29.7	0.2 (0.62)	<0.1 (0.87)
Mean power (% max)	76.3 ± 11.9	77.5 ± 13.8	77.9 ± 6.2	76.7 ± 7.0	<0.1 (0.99)	<0.1 (0.92)
Mean Heart rate (bpm)	158.7 ± 10.3	159.6 ± 7.5	151.0 ± 7.8^#^	147.5 ± 8.1^#^	0.2 (0.64)	13.1 (0.001)
Mean heart rate (% max)^**∗**^	85.4 ± 5.4	84.5 ± 2.7	91.7 ± 4.9^#^	89.1 ± 3.7^#^	1.8 (0.20)	14.6 (<0.001)

^**∗**^Maximum heart rate estimated by the equation: 191.5 − (0.007 × age^2^) [27].

^a^Physical Activity Rating (PA-R) calculated from Jackson Questionnaire [28].

^b^Age-adjusted Fitness Score calculated from Adams and Beam equations [29].

**Table 2:** Exercise-induced changes in NK-cell subset numbers in healthy adult males (*N*_CMV+_ = 20; *N*_CMV−_ = 20) contrasted by CMV serostatus and age. CMV^pos^ and CMV^neg^ participants are denoted by + and −, respectively. Main and interaction effects for CMV, age, and time are reported with significance connoted by ^*∗*^(*p* < 0.05). Statistical differences from pre- and 1 h post-values are described by # and ∧, respectively (*p* < 0.05). Data are mean ± SD.

NK-Cell subsets	CMV status	Pre-values	Post-values	1 h post-values	Main effects *F* statistic (*p* value)			Interactions *F* statistic (*p* value)			
					Time	Age	CMV	Time × Age	Time × CMV	Age × CMV	Time × Age × CMV
Total NK-cells/*μ*L			#∧	#	157.7^*∗*^ (<0.001)	2.6 (0.108)	5.7^*∗*^ (0.019)	0.6 (0.557)	4.7^*∗*^ (0.019)	1.3 (0.252)	1.0 (0.357)
Younger (23–39 yrs)	−	166 ± 96	785 ± 337	130 ± 117							
	+	181 ± 97	595 ± 360	128 ± 84							
Older (50–64 yrs)	−	223 ± 56	987 ± 182	142 ± 57							
	+	189 ± 85	666 ± 242	153 ± 69							
CD56dim (cells/*μ*L)			#∧	#	157.1^*∗*^ (<0.001)	2.8 (0.085)	5.6^*∗*^ (0.020)	0.7 (0.518)	4.7^*∗*^ (0.018)	1.7 (0.197)	1.1 (0.333)
Younger (23–39 yrs)	−	147 ± 91	738 ± 325	106 ± 100							
	+	162 ± 94	556 ± 357	112 ± 82							
Older (50–64 yrs)	−	205 ± 58	942 ± 184	125 ± 57							
	+	176 ± 79	631 ± 217	135 ± 54							
CD56 bright (cells/*μ*L)			#∧		25.2^*∗*^ (<0.001)	1.1 (0.291)	2.5 (0.114)	<0.1 (0.999)	0.4 (0.687)	<0.1 (0.834)	0.5 (0.636)
Younger (23–39 yrs)	−	19 ± 12	47 ± 27	24 ± 22							
	+	19 ± 9	39 ± 15	16 ± 7							
Older (50–64 yrs)	−	18 ± 9	45 ± 23	17 ± 6							
	+	13 ± 10	35 ± 31	18 ± 15							
KLRG1+ (cells/*μ*L)			#∧		72.6^*∗*^ (<0.001)	0.1 (0.773)	2.1 (0.153)	0.1 (0.929)	1.1 (0.335)	0.1 (0.788)	0.1 (0.948)
Younger (23–39 yrs)	−	98 ± 76	493 ± 240	80 ± 73							
	+	84 ± 70	334 ± 284	56 ± 64							
Older (50–64 yrs)	−	111 ± 45	481 ± 149	78 ± 13							
	+	95 ± 64	398 ± 198	69 ± 44							
CD57+ (cells/*μ*L)			#∧		98.5^*∗*^ (<0.001)	5.3^*∗*^ (0.023)	5.2^*∗*^ (0.024)	1.7 (0.196)	2.5 (0.084)	2.7 (0.105)	1.0 (0.360)
Younger (23–39 yrs)	−	63 ± 39	335 ± 190	53 ± 49							
	+	74 ± 48	310 ± 184	50 ± 32							
Older (50–64 yrs)	−	125 ± 29	578 ± 146	87 ± 29							
	+	110 ± 46	453 ± 109	80 ± 29							
CD158a+ (cells/*μ*L)			#∧		50.7^*∗*^ (<0.001)	0.9 (0.349)	2.7 (0.103)	0.3 (0.717)	1.3 (0.284)	0.2 (0.698)	<0.1 (0.980)
Younger (23–39 yrs)	−	40 ± 25	228 ± 191	31 ± 34							
	+	40 ± 20	179 ± 87	28 ± 19							
Older (50-64 yrs)	−	51 ± 37	277 ± 91	32 ± 28							
	+	25 ± 16	119 ± 97	17 ± 15							
CD8+ (cells/*μ*L)			#∧		79.4^*∗*^ (<0.001)	8.4^*∗*^ (0.004)	1.2 (0.269)	2.7 (0.069)	1.7 (0.193)	4.8^*∗*^ (0.031)	3.0 (0.052)
Younger (23–39 yrs)	−	51 ± 35	184 ± 126	45 ± 46							
	+	61 ± 37	210 ± 94	42 ± 28							
Older (50–64 yrs)	−	94 ± 36	406 ± 159	62 ± 21							
	+	62 ± 43	200 ± 75	39 ± 22							
